The article "Supervision and Assistance Based on Mobile Information System in Art Video Teaching" was retracted in 2023. Reasons: suspected computer-generated content; unreliable results or conclusions; concerns about the data; concerns about the results or conclusions.

# Supervision and Assistance Based on Mobile Information System in Art Video Teaching

**DOI:** 10.1155/2022/4658975

**Published:** 2022-06-24

**Authors:** Yang Shi

**Affiliations:** Fine Arts Academy, Changchun Normal University, Changchun 130000, Jilin, China

## Abstract

To enrich students' learning methods, improve their interest in learning, and enable students to fully understand and master the content of art video teaching, a supervision and assistance function based on mobile information system in art video teaching is proposed. Starting with the purpose of improving the auxiliary effect of art video teaching, this study deeply discusses the construction of personalized art video mobile information teaching system based on mobile information technologies such as self-media auxiliary technology and computer-aided technology. Therefore, this study takes android technology mobile information system as a breakthrough to design the video teaching system and introduces the design of mobile teaching information platform in detail. At the same time, according to the relevant requirements of art video teaching, this study designs the teaching system from the aspects of improving students' learning interest, promoting students' curriculum preference information, efficient real-time teacher-student interaction, and so on. According to the requirements of the six sections, the function of the teaching supervision and management module is improved. Through the test of result extraction and data analysis, the feasibility of the user preference extraction and analysis algorithm and the content similarity discrimination algorithm is finally verified. The results show that after more than 10 times of reading, the graphics of video teaching content can basically solve the problem of comparative similarity of the same type of teaching content. At the same time, after more than 30 times of reading, the teaching content can basically solve the problem of small probability error of user system.

## 1. Introduction

At a time when science and technology are advancing rapidly, education reform needs to be deepened. The introduction of multimedia technology in the classroom is an important part of education reform. Demonstration not only stimulates students' interest in learning but also helps them to understand and master the content of art video training and to compensate for the intuition, three-dimensional senses, and deficiencies of traditional teaching methods. It also breaks the boundaries of time and space and creates an open environment for teaching, so that it is possible to implement teaching activities in the form of individual training [1]. The current situation of multimedia-assisted art video teaching is reexamined in recent years and has a more clear and profound understanding of multimedia teaching. It is clear that multimedia, as a modern teaching organization form, is of great significance to improve teaching quality and students' comprehensive quality and teachers' teaching level [2, 3]. Using multimedia to organize teaching is not only to improve the teaching effect but also to realize individual teaching and advocate the teaching form of “individualization,” which is not to cancel or replace the traditional teaching organization form [4]. Its essence is to try to realize the supplement and benefit of “individualization” and “collectivization,” so as to fill the serious defects of the uniformity and rigidity of traditional classroom teaching. Art video teaching mostly focuses on “individualized” teaching, and multimedia teaching organization form can just implement individualized teaching [5].

The article "Supervision and Assistance Based on Mobile Information System in Art Video Teaching" was retracted in 2023. Reasons: suspected computer-generated content; unreliable results or conclusions; concerns about the data; concerns about the results or conclusions.

The information technology skills needed for modern social life are adapted, and the information literacy and the awareness of technological innovation are consolidated. Therefore, it can be seen that this course occupies an important position in the field of education and has far-reaching implications and influence on students' learning and life development. The education of junior high school information technology course has also become a very important link in the process of students' learning and development. The Internet has basically achieved deep penetration in China. In this regard, China is ahead of the world, and this penetration rate is still maintaining a rapid upward development trend. Based on this good situation, we can find that people's daily dependence on life and work and learning TikTok are increasing and the popularity of mobile Internet is increasing. The contact and demand for information also increase, and the way to get information is more and more abundant, for example, microblog, WeChat, and jitter [6]. The birth of these We Media has expanded the access to information. In the powerful network environment, it greatly improves the convenience of using We Media, especially students, who have strong adaptability to novelty. After the emergence of this new media form, it immediately attracts students' attention and changes their learning methods. It is understood that We Media has entered the classroom of primary and secondary schools, covering many disciplines such as language and number. Due to the specifics of the science of art, the introduction of the media in the field of art meets the requirements of the development of the information age. China itself has entered the media era, and there is an urgent need to explore new methods of teaching art video. However, how to make full use of modern technology and better develop art video lessons has not received enough attention from researchers [7]. This study aimed to explore the use of the advantages of We Media for auxiliary teaching, so that students and teachers are not limited by class time and place in learning and communication and carry out more in-depth and directional learning with students with the help and guidance of teachers, to enable them to actively invest in art classes.  Figure 1 is an architectural design diagram of the mobile Internet age information system. In the real-world learning process, students can take full advantage of the convenience and speed of independent media and fully participate in their own subjective initiatives to facilitate the learning process. Teachers benefit from the vividness and directness of We Media, the teaching methods and contents become diversified, and they will be more handy in the process of practice. The quality of the classroom and the overall teaching efficiency will also be improved. Self-media integrated teaching not only is an effective solution to the relevant problems in the current art video teaching practice in junior middle school but also can provide a better platform and carrier for teaching activities and students' autonomous learning [8].

The article "Supervision and Assistance Based on Mobile Information System in Art Video Teaching" was retracted in 2023. Reasons: suspected computer-generated content; unreliable results or conclusions; concerns about the data; concerns about the results or conclusions.

## 2. Literature Review

The United States, Britain, Germany, Japan, Canada, and many other developed countries have already used multimedia to assist art video teaching. As early as the beginning of the century, the United States showed such a development clue of multimedia teaching technology as “visual teaching-audio-visual teaching-teaching media-audio-visual communication” [9]. The use of systematic and reasonable integration methods is the core and soul of art education in the pursuit of optimizing teaching effect. When it comes to the production and use of educational media, it summarizes 12 principles, of which three principles are particularly emphasized: first, if the effect of teachers' teaching and using media is the same, media should not be used; second, the purpose of using teaching media is to teach students, not to shine; and third, if you use low-value teaching tools and high price teaching tools, the effect is as good as that. Do not use high price ones. Many schools have begun to use self-media to organize teaching [10]. Taking the United States as an example, they not only have a wide variety of We Media but also have a wide range of popularization and application. They have not only been recognized by the people but also promoted the teaching reform. Teachers can consciously and flexibly use self-media and perfectly combine it with practical teaching, which promotes the further improvement of teachers' own ability and teaching quality. It can be seen that education in Western countries has more advanced technology and more mature platform, which provides a good case for this study [11]. From the perspective of China, the application of We Media in art video teaching is still in a low stage and lacks deeper exploration and research. The existing problems are mainly reflected in: first, the attention to We Media is not enough; second, the promotion of new forms takes some time. Today, We Media live teaching has been deeply recognized by the majority of people. I believe that soon the application of We Media to auxiliary art video teaching can also be popularized and become an important form of art video teaching [12].

The article "Supervision and Assistance Based on Mobile Information System in Art Video Teaching" was retracted in 2023. Reasons: suspected computer-generated content; unreliable results or conclusions; concerns about the data; concerns about the results or conclusions.

In China, the practice and research of multimedia teaching are far behind the world development level compared with the developed countries in the world. In modern times, multimedia teaching has gradually developed. The important role of multimedia teaching began to be realized by many schools and teachers, and multimedia teaching was taken as the main research direction of teaching and research, and it was also introduced into the teaching of various disciplines. When talking about the future teaching, it was generally believed that individualization has become one of the directions of teaching development due to the development of technology [13]. Some scholars have also made positive affirmation on the significance and advantages of multimedia teaching and put forward some problems that need attention on the integration of multimedia and art [14]. Some scholars talked about the transformation of the organizational form of art video teaching—from class teaching to the coexistence of various teaching forms. On the one hand, this transformation will take into account the individual differences in students and allow students to selectively accept their insufficient and needed knowledge and skills in autonomous learning. At the same time, it fundamentally ensures that the necessary and individualized creativity of art students can be publicized to the greatest extent in diversified teaching forms. Although there are many people studying multimedia-assisted instruction, most of them praise the advantages of multimedia, while few study its disadvantages, and most of them just stay on the surface [15].

## 3. Research Methods

### 3.1. Teaching Platform Design of Mobile Information Function System Based on Android

#### 3.1.1. Design of Information Push Function of Mobile Teaching Platform

The information push function of this platform is mainly to solve how to provide students with the required news content. The news content pushed to the students is obtained through the network, screened and classified by professionals around the cadre education and training content, and finally pushed to the students who need it. In this process, two problems need to be solved: one is how to extract the characteristics of students' interest and news content and establish the measurement standard of the relationship between them; the second is how to push the news information of interest to the mobile terminal by the server. Therefore, two technical details are involved: student interest extraction and information push platform construction.

*(1) User Preference Extraction and Analysis*. User preference extraction and analysis technology is a technology to determine user preferences through the analysis of users' network behavior in the process of using network information resources [16]. Its network behavior includes inquiry, browsing, attention, collection, and evaluation of relevant resources. Through the collection and summary of this information, an analysis model is established to mine the corresponding data, so as to obtain user preferences and save them as user information, so as to provide basic data for deeper information services [17]. The corresponding attributes of resources are given by labeling them. The user's preferences and needs are determined through the user's search behavior. Tag-based preference analysis is mainly divided into three categories: user common tag analysis, which marks different attributes of users through tags, finds the tag coincidence degree between users, infers the user interest similarity based on this, and classifies users; resource tag group analysis is to connect through user tags and tags of resources selected by users; that is, tag resources with user tags to mine information that can be pushed to users. According to the analysis of common tags, because there are multiple tags in a resource, when users access the resource, the tag of the resource is associated with the user. When users have common resource tags and user tags in the system, there will be a strong connection between the common tags [18].

*(2) Information Push Design of Mobile Teaching Platform*. Information push technology is a kind of technology that the computer system infers, perceives, and excavates the user's thinking by analyzing the user's behavior, obtains the characteristics of the user's needs, collects the relevant information of the needs through the intelligent network, and finally transmits it to the user in an appropriate way [19]. The working process of information push is divided into three levels: one is the user information base, which not only records the user's information but also records the user's behavior, to confirm the user's needs; the second is to establish a knowledge base, through the data mining of the server database, establish a knowledge base to record the characteristics of users and information association, and accumulate a knowledge model; and the third is the information push mode of the push server, which obtains the information delivery needs of different users through analysis, such as push time, push mode, total amount, and frequency of distribution. Common classic push mechanisms include android cloud-to-device messaging (C2DM), message queuing telemetry transport (MQTT), the extensible messaging and presence protocol (XMPP), and communication protocol based on XML protocol.

*(3) Construction of Information Promotion Platform*. After in-depth research on information push technology and combined with the actual development of the platform, it is decided to adopt Apache server, Linux system, MySQL database, and LAMJ architecture of JSP, which is relatively suitable for mobile application information push, and run the communication protocol scheme based on XML protocol. According to the application requirements of the teaching information platform of the party school, the push mode combining push and pull is adopted.

*(4) User Interest and News Information Push Model Design*. By analyzing the relationship between users and news, we can find that when users choose news, news is labeled with a certain label, which can reflect the characteristics of news to some extent. At the same time, the selected news also carries out corresponding annotation for user preference characteristics. In this way, users read a large number of interesting news, and their preference characteristics are more obvious. The actual teaching situation of cadre training in party schools is different from that in general education colleges, and the teaching cycle of each shift is generally one and a half months. About 3000 trainees can be trained every year. Students need to learn a lot of training content during school, so the number of news browsing will be greatly limited. Moreover, the news pushed by the teaching information platform is strictly screened and classified, which will be very different from the professional news client in quantity. Therefore, the news information push model of the platform needs to quickly establish the relationship between users and news in a limited time and a small amount of information and data environment. For the above special reasons, this study makes corresponding trade-offs for the description of users and news features [20, 21].

The article "Supervision and Assistance Based on Mobile Information System in Art Video Teaching" was retracted in 2023. Reasons: suspected computer-generated content; unreliable results or conclusions; concerns about the data; concerns about the results or conclusions.

### 3.2. User Preference Extraction and Analysis Algorithm

#### 3.2.1. Selection of User Preference Extraction and Analysis Algorithm

Algorithms for extracting and analyzing user preferences are mainly used to create a model to analyze user preferences, to calculate the weight of user choices in the model as a test point for customer preferences, or to extract a large number of user behavior data. Data and basic signal extraction methods include RSS technology, clustering, genetic algorithms, *k*-means algorithms, or the creation of a rough set decision table. At the same time, the effects of time forgetting parameters and the introduction of long-term and short-term interest parameters are taken into account. Combined with the actual design of the platform, due to the relatively short training and learning time of party school cadres and the annual training volume of about 3000 trainees, the data information generated on the platform is relatively limited. Therefore, the scheme of extracting user preferences based on a large number of data mining will affect the accuracy of information extraction due to the limitation of the amount of data. The construction of rough set decision table is mainly aimed at the extraction of user interest features in incomplete information system. The mobile teaching information platform of the party school is relatively simple, but the system structure is complete, so the rough set decision table is not suitable for the situation of the party school [22]. Due to the limitation of the training time of party school cadres, the influence of long-term and short-term forgetting parameters and time forgetting parameters on interest transfer and extraction is relatively weak, which can be ignored, transferred, or weakened. To sum up, the user preference analysis algorithm most suitable for the teaching environment of the party school should rely on the way of weight calculation.

#### 3.2.2. Design of User Preference Extraction and Analysis Algorithm Based on Weight Plunder

Users' speed of reading news content varies from person to person, but as far as I am concerned, the speed of reading a news is roughly the same, which is determined by users' personal habits. However, users will pay more attention to the content they are interested in than under normal conditions and will think and analyze the corresponding content when reading. It is directly reflected in the decline of reading speed caused by thinking; that is, the time spent reading articles of the same length will be relatively longer. It can be seen that when users read the content they are interested in, the degree of interest is inversely proportional to the reading speed. This platform should be based on a model of algorithmic analysis of consumer preferences based on weight loss and should be able to quickly reflect the characteristics of consumer preferences in a relatively short period of time according to the application of the party's school training platform. During reading, the characteristics of the user's interest change continuously during the reading, gradually approaching the basic characteristics of the user. While reviewing the headline, the user clicks on the headline to enter the detailed viewing interface, and after viewing the headline for a specified period of time, the user is considered interested in the headline [23]. Then, *G*_*ij*_=1 is set to indicate that user I is interested in news *J*, and *G*_*ij*_=0 indicates that user *I* is not interested. The speed of users' browsing news reflects users' attention to this kind of news. Size is the total number of words read by the user, and time is the total time consumed in reading. The average reading speed of user is set as *I*, as shown in the following equation:

(1) $$\begin{array}{c} V_{\text{i}}=\frac{\text{Sina}\left(i\right)}{\text{time}\left(i\right)}. \end{array}$$

When formula (2) is satisfied:

(2) $$\begin{array}{c} t_{\min}\leq t_{\left(ij\right)}\leq 2\frac{\text{Sine}\left(j\right)}{V_{i}}. \end{array}$$

The reading speed of user *i* to news *j* can be expressed by the following formula:

(3) $$\begin{array}{c} s=\frac{\text{Sina}\left(i\right)}{\text{time}\left(ij\right)}. \end{array}$$

At the same time, it can be concluded that the degree of concern of user *i* to news *j* is shown in the following formula:

(4) $$\begin{array}{c} Z_{ij}=\frac{V_{i}}{V_{ij}}. \end{array}$$

When the actual reading time meets the requirements of the following formula:

(5) $$\begin{array}{c} {\text{time}}_{\left(ij\right)}\geq 2\frac{\text{Sine}\left(j\right)}{V_{i}}. \end{array}$$

It indicates that the user has read for a long time or left after reading, and it is determined that the user is interested in the news and pays attention *Z*_*ij*_=2. When the actual reading time (*ij*) is less than *t*_min_, it is considered that the user is not interested in the news and quits before browsing, and the attention is 0.

The article "Supervision and Assistance Based on Mobile Information System in Art Video Teaching" was retracted in 2023. Reasons: suspected computer-generated content; unreliable results or conclusions; concerns about the data; concerns about the results or conclusions.

The interest of end users in news is shown in the following formula:

(6) $$\begin{array}{c} X_{ij}=G_{ij}\times Z_{ij}. \end{array}$$

The user's interest characteristics can be marked by the accessed news content attributes; that is, each time a news is accessed, the user's interest model state will change. The user's interest model can be divided into explicit and implicit parts, which, respectively, correspond to the user's interests (economy, politics, culture, society, etc.) and the implicit corresponding to the initial parameter setting of news attributes (philosophy, science and society, agriculture, science and technology, etc.). The user's interest model is represented by the weight values of explicit and implicit parameters. When the user initially registers and selects all or no interest options, the weight of each interest option is the average value of 0.1, as shown in Table 1.

The reason for the weight change is the change in feedback after viewing the data, and the criterion for the selected option is the sum of the weights of the unselected option if its single value is greater than the mean.

The plunder coefficient formula is as follows:

(7) $$\begin{array}{c} \alpha =\frac{\sum W_{T}}{\sum W_{F}}. \end{array}$$

When 0.1 ≤ *α* ≤ 10, the weight ratio is as follows:

(8) $$\begin{array}{c} \beta =\frac{1}{100\alpha }. \end{array}$$

When *α* < 0.1, the weight ratio is *β* = 0.1, and when *α* > 10, the weight ratio is *β* = 0.

For the process of weight plundering, firstly, the interest options are divided into two categories, and the weights are summed, respectively; the weight formula is applied; and then, the sum of the weights from the selected option to the unselected option is as follows:

(9) $$\begin{array}{c} \varepsilon =\sum W_{F}\times \beta . \end{array}$$

Assuming that the option is selected in I, the weight is obtained for each selected option *ε*/*i*, and each unselected option loses its weight *ε*/(10 − *i*). For example, the initial registration of users selects economy, politics, and culture. Then, the weight changes to

(10) $$\begin{array}{c} \alpha =\frac{0.1\times 3}{0.1\times 7}=0.429,\\ \beta =\frac{1}{100\alpha }=0.023,\\ \varepsilon =0.1\times 7\times 0.023=0.016. \end{array}$$

The weight changes after the user's initial interest selection are shown in Table 2.

When the reason for the weight change is the feedback change after browsing the news, and the judgment standard of the selected option is that its single value is greater than the average value, the sum of the weight of the selected option to the unselected option is shown in the following equation:

(11) $$\begin{array}{c} \varepsilon^{\prime }=X_{ij}\sum W_{F}\times \beta . \end{array}$$

Similarly, the same calculation method is used for the user's implicit preference parameters. When the weight value of the plundered interest item is 0, the weight that should be deprived is shared equally by other unselected interests. The characteristic of this algorithm is to judge whether a user is interested in a certain content, and it does not need how high the weight of the interested option is, as long as it is higher than the average value [24].

The article "Supervision and Assistance Based on Mobile Information System in Art Video Teaching" was retracted in 2023. Reasons: suspected computer-generated content; unreliable results or conclusions; concerns about the data; concerns about the results or conclusions.

#### 3.2.3. Design of News Feature Model

The news information on the mobile teaching platform is captured by the network crawling tool on the subchannel of the special website. The captured data are stored in the preselected database, screened by teachers or educational administrators with senior theoretical basis, and stored in the database after marking the news category and news attribute parameters. The news category setting is equivalent to the user's initial interests and hobbies, and the news attribute parameters are cataloged with reference to the ODP classification principle. The initial parameters of news implicit attribute are as follows: philosophy, science and society, agriculture, science and technology, management, information technology, cadre quality, Marxism, personal charm, and anti-corruption. The weight change in the news feature model does not need to consider the time factor. The sum of the weight plundered from the selected option to the unselected option is shown in the following formula:

(12) $$\begin{array}{c} \varepsilon =\sum W_{F}\times \beta . \end{array}$$

Through the above research, the expression method of user preferences and news features adopts the way of vector space model. Because the definition content of user preferences and news feature vector space is the same, there is no need to make corresponding conversion, and only the explicit characteristics and implicit characteristics need to be calculated separately. The user preference feature vector is as follows:

(13) $$\begin{array}{c} U=\left\{W_{1};W_{2}\text{…}W_{10}\right\}. \end{array}$$

The news feature vector is as follows:

(14) $$\begin{array}{c} N=\left\{NW_{1};NW_{2}\text{…}NW_{10}\right\}. \end{array}$$

The matching degree between news and user interests can be obtained by cosine similarity calculation. The similarity calculation is shown in the following equation:

(15) $$\begin{array}{c} \cos\left(U,N\right)=\frac{\sum_{i=1}^{10}\sum_{j=1}^{10}W_{i}\times NW_{j}}{\sqrt{\sum_{i=1}^{10}W_{i}^{2}\sum_{j=1}^{10}NW_{j}^{2}}}. \end{array}$$

In vector matching, explicit vector and implicit vector are calculated separately. When information is pushed and selected, any vector standard approximation can be regarded as similarity matching. The user's implicit vector parameters can be used as an important basis for the course push of video information resources. The similarity algorithm between individuals suitable for calculating symbolic measure or Boolean measure is referred: “Tanimoto coefficient-based similarity” to design the similarity discrimination algorithm of user's simple preference news. That is, the relationship between users' simple preferences and the attribute characteristics of news is the relationship between sets. We need to judge the relationship between users and news by discussing the relationship between intersection and union between sets. The details are shown in the following formula:

(16) $$\begin{array}{c} \sin\left(U,N\right)=\frac{n_{\text{user}}\cap n_{\text{news}}}{n_{\text{user}}\cup n_{\text{news}}}. \end{array}$$

The screening criteria for information push are divided into several levels.

The article "Supervision and Assistance Based on Mobile Information System in Art Video Teaching" was retracted in 2023. Reasons: suspected computer-generated content; unreliable results or conclusions; concerns about the data; concerns about the results or conclusions.

Cosine Similarity Calculation: it includes explicit and implicit similarity. If both meet, it is accurate similarity, and if one meets, it is relatively accurate similarity. Comparison of Simple Preference Options: it includes the comparison of explicit and implicit simple preference options. If both meet, it is simple and accurate similarity, and if one meets, it is relatively simple and accurate similarity. Cosine similarity is more accurate than simple preference similarity comparison. However, users' simple preference news similarity discrimination is based on the absolute judgment of common interest attributes, that is, yes or no judgment, so its implementation strategy in the process of news discrimination and screening is more rigorous. In the process of information screening, if there are too few relevant resources, the simple preference similarity distinction can be temporarily abandoned and the cosine similarity can be determined directly.

## 4. Results and Discussion

### 4.1. User Interest Model Hobby Extraction and Analysis Algorithm Test

Test Method: the operation rules of user interest extraction model are constructed through the simulator, and targeted test case data are set according to different test contents. The test case data are input into the model, the test data of each case are obtained and a table is formed, the table is analyzed and compared, and the operation law of the data is summarized, to judge the application characteristics of the model, compare the expected effect of the model, and find the gap. Test Premise Constraints: when the weight of the user's interest point is greater than the average value of the overall weight of 0.1, this interest point is the user's characteristic interest, which is different from the user's general interest. The selected interest point is the feature of the news read by the user or the interest feature selected by the user [25]. The test purpose is divided into two parts, including that the model can reflect the user's interest and realize the correctness of interest extraction; the model can distinguish the correctness of interested news according to user interest. Test Process of Test: the simulator is used to construct the user interest model, the test cases are set according to the test steps, the complexity of the test cases is gradually increased from shallow to deep, the characteristics of the results of each test case are gradually analyzed and summarized, and the final conclusion is formed.

The article "Supervision and Assistance Based on Mobile Information System in Art Video Teaching" was retracted in 2023. Reasons: suspected computer-generated content; unreliable results or conclusions; concerns about the data; concerns about the results or conclusions.

#### 4.1.1. The Interest Points of the Test Model Tend to Balance with the Increase in Reading

Case Name: It is stability test of model feature points of interest.

Use Case Function Description: it tests whether the weight of interest points tends to be stable when the model reads a large number of similar news.

Use Case Content Description: 50 news items are input including economic, political, and cultural categories into the model.

Expected Result of Use Case: the weight of the selected interest point gradually increases with the amount of news reading and vice versa.

The test data results are shown in Figures 2–4.

Graphic Data Analysis: it can be found from Figure 4 that with the continuous rise of individual weights of user characteristic interest points, the curve is gradually flattened, and the effect of plundering weights from general interest points is gradually weakened. When reading a kind of news for more than 30 times, the change in weights tends to be stable. It can be seen that when users browse the news, the weight corresponding to the user's preference characteristics will gradually change with the different news they browse. Because users choose based on their personal preferences in the process of reading the news, the change in this weight will reflect the user's interest characteristics. Analysis Conclusion: the test effect meets the design expectation. This algorithm has personal preferences, and the content of reading news is changing at will. According to the convergence of graphics, this algorithm has the characteristics that the larger the number of news users read, the more they can reflect their reading characteristics and makes the user's preference characteristics stable.

#### 4.1.2. The Test Model Has the Characteristics of Protecting the Original Interest

Expected Result of Use Case: after reading the news for 25 times, the selected interest points become unselected interest points. The weight of the original feature points of interest decreases gradually with the amount of news reading, but the final weight is still higher than the average value. The test data results are shown in Figures 5–7.

Graphic Data Analysis: this use case has certain reverse interference characteristics. Through Figure 5, it can be found that the weight change in the user's original feature interest finally stays above 0.1, and the weight of the general interest point does not exceed 0.1, indicating that the model has certain protection against the reduction in the feature interest weight when the user's original feature interest point is disturbed by other interest points. The reading amount of interest points fluctuated with the reading amount at the 25th time, but the overall trend was still gradually stable. It shows that the model can still highlight the user's original characteristic interest in the case of reverse interest point interference.

The article "Supervision and Assistance Based on Mobile Information System in Art Video Teaching" was retracted in 2023. Reasons: suspected computer-generated content; unreliable results or conclusions; concerns about the data; concerns about the results or conclusions.

Analysis Conclusion: the test results meet the design expectations, indicating that the model has the characteristics of protecting the original interest.

#### 4.1.3. Testing Models Can Generate New Interest

Description of Use Case Content: 30 news including economic, political, and cultural categories are input into the model, and then, 20 news of political, cultural, and social categories are input into the model (remove economy and increase society). Expected Result of Use Case: after reading the news for 30 times, the weight of economic interest points gradually decreases and the weight of social interest points gradually increases. After a certain amount of reading, the weight is greater than the average value of 0.1. The test data results are shown in Figures 8–12.

Analysis Conclusion: it is in line with the expectation. The model supports the generation of new feature interest. At the same time, the proof algorithm has a protective effect on specialty interest. The greater the amount of reading, the better it can reflect the user characteristics.

#### 4.1.4. Functional Test of Distinguishing Different Types of News

Use Case Name: different kinds of news function test news use case function description are distinguished: whether the module can distinguish the distance between news and user interest when inputting different kinds of news is tested. Use Case Content Description: an economic, political, and cultural news and a legal, international, educational, and military news are input into the model, respectively, to compare the similarity with the user interest use case, as shown in Figure 13.

Graphic Data Analysis: it can be found in Figure 13 that with the increase in users' reading, the distinction between the two lines becomes larger and larger, and similar news is obviously at the top. It can be seen that the distinction between news models with different feature classifications is more obvious. Analysis Conclusion: the model has the function of distinguishing different kinds of news.

The article "Supervision and Assistance Based on Mobile Information System in Art Video Teaching" was retracted in 2023. Reasons: suspected computer-generated content; unreliable results or conclusions; concerns about the data; concerns about the results or conclusions.

## 5. Conclusion

Nowadays, the personalized development needs of student education are becoming more and more prominent, and the traditional teaching mode should be innovated accordingly. The teaching mode studied in this study is based on the emerging media of “We Media.” The modern educational technology is combined with traditional teaching mode, the methods and means of applying it to art video teaching are explored, and the theory and practice of current education are combined, to build a personalized, free learning, and better experiential efficient teaching mode, to make the form of art education more diversified. This study designs the art video teaching information platform based on android mobile intelligent terminal in detail and focuses on the design of preference analysis information push, efficient real-time teacher-student interaction, and other contents. The function realization effect involved in these research contents is the embodiment of the essential difference between this platform and the traditional teaching information platform. At the same time, other functional modules to realize the overall function of the platform are designed accordingly, and the system operation mechanism in the process of realizing the functions of relevant modules is deeply studied. Finally, it realizes the relevant functions of the six sections of ordinary users of the platform and the simple management module of teachers. At the end of the study, by simulating the actual environment and using the test steps of use case input, result extraction and data analysis, the feasibility and superiority of user preference extraction, and analysis algorithm and news similarity discrimination algorithm are verified.

## Figures and Tables

**Figure 1:** Architecture design and technical implementation of information system in the era of mobile Internet.

**Figure 2:** Changes in individual weights of user interest points with reading volume.

**Figure 3:** Changes in individual weights of users' noninterest points with reading volume.

**Figure 4:** Variation of plunder volume with reading volume.

**Figure 5:** Changes in users' original interest points.

**Figure 6:** Changes in original noninterest points of users.

**Figure 7:** Variation of plunder volume with reading volume.

**Figure 8:** Changes in original noninterest points of users.

**Figure 9:** Changes in new user interest points.

**Figure 10:** Changes in users' original interest points.

**Figure 11:** Users' original interest points become noninterest points.

**Figure 12:** Variation of plunder volume with reading volume.

**Figure 13:** Comparison and similarity of different types of news.

The article "Supervision and Assistance Based on Mobile Information System in Art Video Teaching" was retracted in 2023. Reasons: suspected computer-generated content; unreliable results or conclusions; concerns about the data; concerns about the results or conclusions.

**Table 1:** User initial weights.

	Economics	Politics	Culture	Sociology	Law	International	Education	Military	Ecology	Party building

Weight	0.100	0.100	0.100	0.100	0.100	0.100	0.100	0.100	0.100	0.100

**Table 2:** Weight after user interest selection.

	Economics	Politics	Culture	Sociology	Law	International	Education	Military	Ecology	Party building

Weight	0.105	0.105	0.105	0.097	0.097	0.097	0.097	0.097	0.097	0.097

## Data Availability

No data were used to support this study.
